# Expression of Adenosine Deaminase and NLRP3 Inflammasome in Tuberculous Peritonitis and Their Relationship with Clinical Efficacy

**DOI:** 10.1155/2022/3664931

**Published:** 2022-09-15

**Authors:** Hongwei Su, Guorong Yan, Zijian Li, Lin Fu, Lingdi Li

**Affiliations:** ^1^The Second Department of Thoracic Surgery, Hebei Chest Hospital, Shijiazhuang 050040, Hebei, China; ^2^Department of Orthopedics, Hebei Chest Hospital, Shijiazhuang 050040, Hebei, China

## Abstract

**Objective:**

Tuberculous peritonitis (TP) can cause multiple infections of surrounding organs and tissues, leading to organ failure and endangering life safety. In this research, the relationship between adenosine deaminase (ADA), NLRP3 inflammasome, and TP and its clinical significance will be deeply explored, so as to provide new directions and reliable reference opinions for future clinical diagnosis and treatment.

**Methods:**

Altogether, 59 TP patients (research group, RG) and 52 non-TP patients (control group, CG) who were admitted to our hospital from May 2014 to June 2018 were regarded as research objects. Ascites samples of RG before treatment (admission) and one month after treatment and CG before treatment were obtained, and the ADA and NLRP3 levels were tested to evaluate the clinical and prognostic significance of the two in TP.

**Results:**

Before treatment, ADA and NLRP3 in RG were higher than CG (*P* < 0.05), and the sensitivity and specificity of combined detection of the two in predicting TP occurrence were 89.83% and 73.08% (*P* < 0.05). In addition, ADA and NLRP3 in RG patients were positively correlated with the disappearance time of abdominal pain and ascites (*P* < 0.05) and had excellent predictive effect on the adverse reactions during treatment (*P* < 0.05). After treatment, both in RG patients decreased, which was inversely proportional to the clinical efficacy (*P* < 0.05). Prognostic follow-up manifested that ADA and NLRP3 in relapse patients were higher than those without recurrence after treatment (*P* < 0.05).

**Conclusion:**

The increase of ADA and NLRP3 in TP is relevant to the adverse reactions during treatment, clinical efficacy, and prognosis recurrence after treatment. It can be used as a disease marker to confirm, intervene, and evaluate TP progression promptly.

## 1. Introduction

Tuberculous peritonitis (TP) is a chronic and diffuse inflammation of peritoneum caused by mycobacterium tuberculosis, which is familiar in young and middle-aged women, and has a certain potential risk in any age group [1]. According to the survey, there are more than 500,000 new TP patients worldwide every year, 6-8 times higher than that in 2010, which is also relevant to the changes of people's eating habits and living environment [2]. The occurrence of TP can cause multiple infections of surrounding organs and tissues, resulting in organ failure and endangering life safety [3]. In clinical practice, conservative treatment schemes can usually achieve ideal results for early TP; but most patients have no special clinical symptoms in the early stage and may only show intermittent abdominal pain, diarrhea, etc., and they often miss the best treatment period due to lack of medical and health knowledge [4, 5]. For those with severe illness and complicated infection, surgical treatment is needed [6]. At this time, patients may not only need to remove the diseased bowel segment but also need to receive long rehabilitation and antituberculosis treatment after operation, which seriously reduces the quality of life of prognosis [7]. Thus, early detection and treatment of TP are the key to ensure patients' health. At the moment, the differential diagnosis of TP needs a series of blood routine, imaging routine, tuberculin, T-cell spot test, laparoscopy, etc., and the only diagnostic gold standard is peritoneal pathological biopsy [8]. The main reason for the poor prognosis of TP is that early TP has strong concealment, and on the other hand, the examination methods are still complicated, which cannot quickly and accurately evaluate its occurrence and development [9]. Thus, researchers are constantly trying to find a new and reliable TP evaluation method to ensure the treatment effect and prognosis of patients.

Adenosine deaminase (ADA), an enzyme involved in purine metabolism, can maintain the development of immune system [10]. Mycobacterium tuberculosis, a common pathogenic bacterium, will never get sick even if it is infected in people with sound immune system, and TP is caused by abnormal immune function of infected people [11]. This suggests that there may be a certain latent relationship between ADA and TP. For instance, Shen et al. found that ADA had a certain diagnostic potential for TP [12], which proves our conjecture. The NLRP3 responds to the stimulation of metabolic stress signals, leading to caspase-1 activation and IL-1 *β* production, which play an important role in a variety of diseases. Secretion of proinflammatory cytokines IL-1*β* and IL-18 induced by activation of NLRP3 inflammasome, as well as pyrodeath, is self-protective measures that help protect the body against exogenous microbial infection and endogenous cellular damage and maintain homeostasis. Meanwhile, NLRP3 inflammasome is also involved in the occurrence and development of diabetes, making clinical symptoms and treatment more complicated, which is one of the possible mechanisms of diabetic cardiomyopathy. Recent studies suggest that NLRP3 inflammasome may be a potential new target for the treatment of diabetes mellitus [13]. ADA and NLRP3 have been proved to have abnormal expression in TP, but their specific clinical significance is still vague.

Accordingly, this research will deeply explore the relationship and clinical significance of ADA, NLRP3, and TP, aiming at providing new directions and reliable reference opinions for future clinical diagnosis and treatment.

## 2. Materials and Methods

### 2.1. Patient Data

Altogether, 59 TP patients (research group, RG) and 52 non-TP patients (control group, CG) who were admitted to our hospital from May 2014 to June 2018 were considered as the research objects in retrospective analysis. All the subjects signed the informed consent form themselves. The protocol of this study is approved by the ethics committee of Hebei Chest Hospital (no. CL2014/44-341).

### 2.2. Inclusion and Exclusion Criteria

RG: inclusion criteria: age > 18 years old; TP was diagnosed by peritoneal biopsy, accompanied by abdominal pain, abdominal distension, ascites, and other clinical symptoms of TP. X-ray revealed increased abdominal density, intestinal adhesions, calcified lymph nodes, or intestinal obstruction; TP conservative treatment after admission; exclusion criteria: patients with other immune system, blood system, and tumor diseases; patients with organ dysfunction or abnormality; pregnant and lactating patients; those who cannot extract ascites after one month of treatment; prognostic follow-up losers; those who did not follow the doctor's advice during treatment. CG: cancer cells existed in ascites, and tumors were confirmed by pathological biopsy; the exclusion criteria are the same as above.

### 2.3. Therapeutic Methods

After admission, TP patients were treated in strict accordance with guidelines. Early patients were given oral administration, and advanced patients were given intravenous administration. Treatment plans were intensive treatment with rifampicin, isoniazid, and pyrazinamide (or ethambutol and streptomycin) for 2-3 months, and continuous treatment with rifampicin and isoniazid for 7-9 months in the consolidation period. For general exudative TP patients, it is necessary to emphasize the whole course of standardized treatment. For adhesive and caseous TP patients, it is certainly worth combining medication and appropriately extending the course of anti-tuberculosis treatment. The prognosis of TP patients was followed up for 2 years in the form of regular hospital review.

### 2.4. Research Samples

Ascites samples of RG before treatment (at admission) and one month after treatment and CG before treatment were obtained. Supernatant was obtained after centrifugation. ADA level was tested by automatic biochemical analyzer (kit purchased from Shanghai Yaji Biotechnology Co., Ltd.), and NLRP3 level was tested by ELISA (kit purchased from Shanghai Jihe Biotechnology Co., Ltd.).

### 2.5. TP Efficacy Evaluation

After 2 months of treatment, the clinical efficacy of TP patients was evaluated [14]. Cured: clinical symptoms such as abdominal distension and pain, disappearance of abdominal tenderness and rebound pain, softness of abdominal muscles, and normal body temperature; markedly effective: clinical symptoms and signs of abdominal tenderness and rebound pain were obviously improved, and most of abdominal effusion was absorbed; effective: clinical symptoms and signs were relieved, and a small amount of ascites was absorbed. Ineffective: clinical symptoms did not meet the above criteria.

## 3. Statistical Methods

SPSS22.0 software was used for statistical analysis. The measurement data were expressed in percentage and assessed via chi-square test. The counting data were expressed by mean ± standard deviation and evaluated through independent sample *t*-test and paired *t*-test. ROC curve was used for prediction analysis, and Pearson and Spearman correlation coefficients were applied to correlation analysis. *P* < 0.05 was regarded to be statistically remarkable.

## 4. Results

### 4.1. Comparison of Clinical Baseline Data

It was found that there was no dramatic difference in clinical baseline data such as age and gender between RG and CG (*P* > 0.05, Table 1), and both groups were comparable.

### 4.2. Comparison of NLRP3 and ADA Levels

ADA in RG before treatment was (26.42 ± 5.72) U/L, higher than CG (*P* < 0.05, Figure 1(a)). NLRP3 in RG before treatment was (94.05 ± 11.82) pg/mL, higher than CG (*P* < 0.05, Figure 1(b)).

### 4.3. Predictive Value of ADA and NLRP3 for TP

ROC curve analysis manifested that when ADA > 20.77 U/L in ascites, the sensitivity and specificity of predicting TP occurrence were 84.75% and 61.54% (*P* < 0.05, Figure 2(a)). When NLRP3 > 87.26 pg/mL, the sensitivity and specificity were 71.19% and 80.77% (*P* < 0.05, Figure 2(b)). The joint formula of ADA and NLRP3, Log (*P*) = −14.679 + 0.185 × ADA + 0.122 × NLRP3, was obtained by binary regression analysis. When Log (*P*) > 0.38, the sensitivity and specificity of the joint detection of ADA and NLRP3 to predict TP occurrence were 89.83% and 73.08% (*P* < 0.05, Figure 2(c)).

### 4.4. Relationship between ADA, NLRP3, and Disappearance Time of Abdominal Pain and Ascites

The disappearance time of abdominal pain and ascites in RG was (13.61 ± 3.62) and (35.02 ± 6.06) days, respectively. Pearson correlation coefficient analysis demonstrated that ADA and NLRP3 were positively correlated with the disappearance time of abdominal pain before treatment (*P* < 0.05, Figures 3(a) and 3(b)) and also positively correlated with the disappearance time of ascites (*P* < 0.05, Figures 3(c) and 3(d)), that is, the higher ADA and NLRP3, the longer the disappearance time of abdominal pain and ascites is.

### 4.5. Relationship between ADA, NLRP3, and Adverse Reactions

During the treatment, 4 patients had mild rash, 2 had abnormal liver function, 5 had vomiting, and the total adverse reaction rate was 18.64%. ADA and NLRP3 in patients with adverse reactions were higher than those without adverse reactions before treatment (*P* < 0.05, Figures 4(a) and 4(b)). ROC analysis manifested that when ADA > 24.30 U/L before treatment, the sensitivity and specificity of predicting adverse reactions in TP patients were 100.0% and 45.83% (*P* < 0.05, Figure 4(c)). When NLRP3 > 90.15 pg/mL, the sensitivity and specificity were 100.0% and 50.00% (*P* < 0.05, Figure 4(d)). Similarly, the joint formula of ADA and NLRP3, Log (*P*) = −24.547 + (−0.782 × ADA) + 0.461 × NLRP3, was obtained by binary regression analysis. When Log (*P*) > 0.18, the sensitivity and specificity of ADA and NLRP3 combined detection to predict adverse reactions were 72.73% and 83.33% (*P* < 0.05, Figure 4(e)).

### 4.6. Relationship between ADA, NLRP3, and Clinical Efficacy

After treatment, ADA and NLRP3 of ascites in RG were lower than those before treatment (*P* < 0.05, Figures 5(a) and 5(b)). The clinical evaluation results manifested that 15 cases were cured, 26 were markedly effective, 6 were effective, and 12 were ineffective. Subsequently, Spearman correlation coefficient analysis found that after treatment, ADA and NLRP3 in RG were negatively correlated with clinical efficacy (*P* < 0.05, Figures 5(c) and 5(d)), that is, the higher ADA and NLRP3 after treatment, the worse the efficacy is.

### 4.7. Relationship between ADA, NLRP3, and TP Prognosis

During the 2-year follow-up, TP recurred in 9 patients, with a total recurrence rate of 15.25%. After treatment, the ADA of relapsed patients after prognosis was higher than that of those without recurrence (*P* < 0.05, Figure 6(a)), and NLRP3 was also higher (*P* < 0.05, Figure 6(b)). Soon afterwards, ROC analysis denoted that when ADA > 23.86 U/L after treatment, the sensitivity and specificity of predicting TP recurrence were 66.675 and 80.00% (*P* < 0.05, Figure 6(c)). When NLRP3 > 78.97 pg/mL, the sensitivity and specificity were 100.0% and 42.00% (*P* < 0.05, Figure 6(d)). The joint formula of ADA and NLRP3 is Log (*P*) = −7.571 + 0.112 × ADA + 0.039 × NLRP3. When Log (*P*) > 0.16, the sensitivity and specificity of the joint detection of ADA and NLRP3 in predicting TP recurrence were 66.67% and 74.00% (*P* < 0.05, Figure 6(e)).

## 5. Discussion

This research is based on the analysis of ADA and NLRP3 that are relevant to immune function and inflammatory response in human body. The purpose is to determine the exact expression and clinical significance of the two in TP. It is found that both of them have excellent evaluation effect in TP, which is quite significant for making new clinical diagnosis and treatment plans. First, the ADA and NLRP3 levels in TP patients and cancerous ascites patients were tested. It showed that ADA and NLRP3 in ascites of TP patients increased, suggesting that they might be involved in disease occurrence and development. In previous studies, we also discovered that ADA and NLRP3 were elevated in liver cirrhosis and gastroenteritis, which was associated with the results of this experiment [14, 15]. It is well known that ADA, as a key enzyme of purine nucleotide metabolism in human body, can catalyze adenine nucleoside to produce inosine, generate hypoxanthine after nucleotide phosphorylase catalysis, and finally oxidized to uric acid and excreted in vitro [16, 17]. ADA is the highest in red blood cells and T lymphocytes, and its activity is directly related to the number and differentiation degree of T cells, while the immunity of tuberculosis is cellular immunity directly mediated by T lymphocytes [18, 19]. Hence, in TP, mycobacterium tuberculosis antigen stimulates the differentiation of T lymphocytes to accelerate, and the number of T lymphocytes will obviously increase, thus causing the increase of ADA. As for NLRP-3 inflammasome, research has confirmed that NLRP-3 can be activated in the case of bacterial infection, promoting the synthesis and secretion of downstream IL-1*β*, IL-18, and other proinflammatory mediators, and then causing extensive tissue damage [20]. Moreover, Yin et al. have verified that in severe acute peritonitis, even if the symptoms of peritonitis are alleviated, the release of proinflammatory factors can still reach several weeks, which continuously potentially affects the shape and function of peritoneum [21]. From this, both are quite essential to TP, but their specific clinical application value still needs to be further explored. Then, we analyzed the prediction effects of ADA and NLRP3 on TP by ROC curve, and the results revealed that both of them showed remarkable effects, and the sensitivity and specificity of combined detection reached 89.83% and 73.08%, respectively. Compared with the current routine clinical detection items, the detection methods of ADA and NLRP3 are more convenient and faster, which can effectively realize the early clinical screening and evaluation and improve the diagnosis rate of early TP. As the collection of ascites samples is still a difficult examination method, it is still one of the key points of follow-up research to determine whether ADA and NLRP3 in blood samples have the same excellent effect as soon as possible. What is more, this research also found that ADA and NLRP3 were directly proportional to the disappearance time of abdominal pain and ascites in TP patients, suggesting that the increased levels are directly related to the pathological manifestations of patients. This has vital reference significance for TP, which still lacks effective and rapid assessment of disease development. More than that, we confirm that ADA and NLRP3 in patients with adverse reactions during the treatment are high, and they also show excellent results in predicting adverse reactions, which further suggests that both have the potential to become clinical evaluation indicators of TP. When the patients are admitted to the hospital, the detection of ADA and NLRP3 not only can initially judge the occurrence of TP but it can evaluate its development, and timely and quickly carry out symptomatic treatment to the more serious patients to ensure the prognosis. Next, we find that after treatment, the ADA and NLRP3 levels in TP patients decrease, and their levels are directly inversely proportional to the clinical efficacy of patients, which confirms the significance of both for evaluation. In the future, we can learn about patients' rehabilitation process in time through the ADA and NLRP3 level changes during treatment and pay attention to TP that is still at a high level after treatment, so as to effectively improve current clinical treatment effect. Not only that, in the follow-up of prognosis, we understand that the increase of levels of ADA and NLRP3 after treatment is relevant to the prognosis review of patients, and we think it is caused by the close relationship between ADA and NLRP3 and human immune function and inflammatory response, once again emphasizing the close potential relationship between them and TP.

Nevertheless, in clinical practice, there are many factors that affect the adverse reactions, clinical efficacy, and prognosis recurrence of TP patients, which may not only play a potential role in ADA and NLRP3. Therefore, we need to expand the research sample size, strictly guarantee the controllable factors of the experiment, and further analyze the results. Moreover, we will confirm the influence mechanism of ADA and NLRP3 on TP through in vitro experiments and help to further confirm the relationship between them.

## 6. Conclusion

The elevation of ADA and NLRP3 in TP is relevant to the adverse reactions during treatment, clinical efficacy, and prognosis recurrence. It can be used as a disease marker to confirm, intervene, and evaluate TP progression promptly.

## Figures and Tables

**Figure 1:** Comparison of ADA and NLRP3 levels. (a) ADA of ascites in RG and CG. (b) NLRP3 of ascites in RG and CG. ^#^*P* < 0.05.

**Figure 2:** Predictive value of ADA and NLRP3 to TP. (a) ROC curve of ADA in ascites to predict TP occurrence. (b) ROC curve of NLRP3 in ascites to predict TP occurrence. (c) ROC curve of ADA and NLRP3 in ascites to predict TP occurrence.

**Figure 3:** Relationship between ADA, NLRP3, and disappearance time of abdominal pain and ascites. (a) Correlation between ADA and disappearance time of abdominal pain before treatment. (b) Correlation between ADA and ascites before treatment. (c) Correlation between NLRP3 and disappearance time of abdominal pain before treatment. (d) Correlation between NLRP3 and ascites before treatment.

**Figure 4:** Relationship between ADA, NLRP3, and adverse reactions (a). Comparison of ADA of patients with and without adverse reactions before treatment. (b) Comparison of NLRP3 of patients with and without adverse reactions before treatment. (c) ROC curve of ADA predicting adverse reactions of TP patients before treatment. (d) ROC curve of NLRP3 predicting adverse reactions of TP patients before treatment. (e) ROC curve of ADA combined with NLRP3 predicting adverse reactions of TP patients before treatment. ^#^*P* < 0.05.

**Figure 5:** Relationship between ADA, NLRP3, and clinical efficacy. (a) Comparison of ADA in RG before and after treatment. (b) Comparison of NLRP3 in RG before and after treatment. (c) Correlation between ADA after treatment and clinical efficacy. (d) Correlation between NLRP3 after treatment and clinical efficacy. ^#^*P* < 0.05.

**Figure 6:** Relationship between ADA, NLRP3, and TP prognosis. (a) Comparison of ADA of patients with recurrence and nonrecurrence after treatment. (b) Comparison of ADA of patients with recurrence and nonrecurrence after treatment. (c) ROC curve of ADA predicting TP recurrence after treatment. (d) ROC curve of NLRP3 predicting TP recurrence after treatment. (e) ROC curve of ADA combined with NLRP3 predicting TP recurrence after treatment. ^#^*P* < 0.05.

**Table 1:** Comparison of clinical baseline data between RG and CG [*n*(%)]/(^−^*χ* ± *s*).

	CG (*n* = 52)	RG (*n* = 59)	Or *tχ*^2^	*P*
Age (years)	43.33 ± 8.88	42.88 ± 7.46	0.290	0.772
BMI (kg/cm^2^)	21.15 ± 3.71	21.68 ± 3.50	0.774	0.441
Gender			0.668	0.414
Male vs. female	14 vs. 38	12 vs. 47		
Marital status			0.308	0.579
Married vs. unmarried	42 vs. 10	50 vs. 9		
Place of residence			0.049	0.825
Urban vs. rural areas	38 vs. 14	42 vs. 17		
Smoking			0.701	0.403
Yes vs. no	18 vs. 34	25 vs. 34		
Drinking			0.122	0.727
Yes vs. no	12 vs. 40	12 vs. 47		
Family medical history			0.290	0.590
Yes vs. no	7 vs. 45	6 vs. 53		
Nationality			1.002	0.317
Han vs. ethnic minorities	50 vs. 2	54 vs. 5		

## Data Availability

The datasets used during the present study are available from the corresponding author upon reasonable request.
